The article "Exploration of Despair Eccentricities Based on Scale Metrics with Feature Sampling Using a Deep Learning Algorithm" was retracted in 2025. Reasons: unreliable results or conclusions; concerns about the results or conclusions; concerns about the citations; concerns about the article.

# Exploration of Despair Eccentricities Based on Scale Metrics with Feature Sampling Using a Deep Learning Algorithm

**DOI:** 10.3390/diagnostics12112844

**Published:** 2022-11-17

**Authors:** Tawfiq Hasanin, Pravin R. Kshirsagar, Hariprasath Manoharan, Sandeep Singh Sengar, Shitharth Selvarajan, Suresh Chandra Satapathy

**Affiliations:** 1 Department of Information Systems, Faculty of Computing and Information Technology, King Abdulaziz University, Jeddah 21589, Saudi Arabia; 2 Department of Artificial Intelligence, G.H Raisoni College of Engineering, Nagpur 440016, India; 3 Department of Electronics and Communication Engineering, Panimalar Engineering College, Chennai 600123, India; 4 Department of Computer Science, Cardiff Metropolitan University, Cardiff CF5 2YB, UK; 5 Department of Computer Science, Kebri Dehar University, Kebri Dehar 001, Ethiopia; 6 School of Computer Engineering, KIIT Deemed to Be University, Bhubaneswar 751024, India

**Keywords:** audio features, mental imbalance, depression prediction, deep learning

## Abstract

The majority of people in the modern biosphere struggle with depression as a result of the coronavirus pandemic’s impact, which has adversely impacted mental health without warning. Even though the majority of individuals are still protected, it is crucial to check for post-corona virus symptoms if someone is feeling a little lethargic. In order to identify the post-coronavirus symptoms and attacks that are present in the human body, the recommended approach is included. When a harmful virus spreads inside a human body, the post-diagnosis symptoms are considerably more dangerous, and if they are not recognised at an early stage, the risks will be increased. Additionally, if the post-symptoms are severe and go untreated, it might harm one’s mental health. In order to prevent someone from succumbing to depression, the technology of audio prediction is employed to recognise all the symptoms and potentially dangerous signs. Different choral characters are used to combine machine-learning algorithms to determine each person’s mental state. Design considerations are made for a separate device that detects audio attribute outputs in order to evaluate the effectiveness of the suggested technique; compared to the previous method, the performance metric is substantially better by roughly 67%.

## 1. Introduction

Mental illness can also contribute to a wide range of physical ailments. Medical research has found numerous autoimmune diseases, but neither a clear cause nor a perfect cure is currently commercially available. Basic disease generation starts with an individual’s cognitive patterns, unresolved grief, past trauma, and the events and circumstances they have gone through. The coronavirus epidemic has had a profound influence on people’s psychological health. Mental health issues are a common issue today that affects everyone. Anxiety and depression disorders, which affect people of all ages, including children and the elderly, are the most common problems. Machine learning is the most popular technique for analysing this kind of data. As changes in mood, emotions, speech, and body language can affect the severity of depression [1], vowel-based depression diagnosis now includes a category for gender-based depression. In several studies for the diagnosis of depression [2], dialogue structures and classifier implementation have been linked in several ways. The majority of people’s propensity toward suicide is caused by depression. Monitoring a person’s current state reveals a lot about them. The significant signs of severe depression include lack of interest and difficulty concentrating, but it can also include headaches and suicidal thoughts, which dramatically push up the mortality toll. Accordingly, it was found that people between the ages of 13 and 20 are the age group where depression is most prevalent. Early identification is, therefore, essential to prevent later problems [3]. Analysis and continual depression monitoring were conducted using a database of speech recordings. 

When a person’s auditory condition is analysed for medical purposes, total mental disease can be diagnosed without any hiccups. Therefore, it is much better to create a system that uses a time-frame windowing technique rather than installing other devices that offer poor accuracy. Estimates can be made from tiny audio samples and separated into several sorts of measures if a deep feature extraction is employed. Moreover, it is crucial to construct a bio-network that can be directly connected to input devices in order to recognise all of an individual’s cognitive features. Therefore, the majority of devices are linked to humanoid intelligence and can track the overall decline in concentration. The lifespan of an individual can be preserved if a decline in concentration is reported to an emergency centre for the necessary action. By providing dialogue at opportune times, the audio depression approach can help many more individuals than the traditional intelligence system. Numerous forms of uncertainty will be a barrier if an audio device is intended to identify a person’s depressed condition [4,5,6,7,8,9,10]. By giving the proper data to all audio devices, which will further decrease functional loss, the problem of uncertainties in the design process will be reduced. More noisy data will be transmitted when there is uncertainty, changing the output properties of the data signal. Furthermore, it becomes considerably more challenging to detect depression using segment design if the computer vision process is sophisticated. Self-trained networks can be used to enable transformation in the automated techniques of diagnosing a person’s mental stress in order to take additional action. Therefore, this study proposes a machine-learning strategy for the speech-based detection of depression. 

### 1.1. Research Gap and Motivation

The major limitation of the existing approach [1,2,3,4,5,6,7,8,9] for identifying the depressed state of an individual is that only wiring-based module components are present; the components are directly connected to display units that provide the state of a person using a three-fold pattern, such as normal, abnormal and indeterminate. However, by using the three-fold pattern, it is not possible to provide quick decisions as the characteristics of an individual are not defined and it is impossible to understand the type of emotional state. Hence to understand the emotional state of an individual, it is essential to have an efficient device that uses appropriate audio inputs for detection. Even some of the traditional approaches [11,12,13,14,15,16,17,18] have incorporated an effective audio monitoring system; however, due to the presence of external noise, the samples are disturbed and the system cannot be operated as a convolutional unit.

Therefore, to observe the characteristics of an individual that are related to a depression state, the proposed method incorporates different audio features. In the first phase of the proposed method, all audio samples are trained using a set of input features and the response that is present at the output fold is measured and stored. In the next phase, some of the time-frame windows are represented for achieving normalised spectrogram values; thus, the frequency values are changed for each interval period. Once the time-frame window is completed, then the deep learning features are added and assimilated in a direct representation form to the designed analytical approach. Hence, at the testing phase for every fold, different metrics are measured, where the accuracy, sensitivity and specificity of the designed audio device are effective, and it is operated within the limited region of the receiver curves.

### 1.2. Paper Organisation

Section 1 is an introduction to the suggested research methodology. A complete literature analysis is included in Section 2 to evaluate the existing methods and approaches for the diagnosis of depression. Section 3 presents the suggested research methodology, while Section 4 presents the findings and recommendations. The results and sources during the research process are expounded upon in Section 5. 

## 2. Literature Survey

Numerous experiments are being done to see whether automated speech analysis can replace the present questionnaire method of diagnosing depression in the presence of mental health professionals. Prosodic, glottal, cepstral, and ethereal acoustic properties have been identified, and they can be divided into two main categories: perceptual (which includes prosodic, spectral, glottal, and cepstral elements) and physiological (which provides for ethereal aspects) (including TEO). The researchers created a standard system architecture to classify sad patients. The Database of Subject’s Speech, the first step in the architecture’s five-step categorisation process, comprises gathering speech samples from healthy and depressed patients to build the database. Preprocessing is another step. The background noise is removed from the audio files in this step, and the audio of the patients and doctors is segregated for feature extraction and analysis. In the extraction stage, various feature extraction techniques are used to extract various components from the speech while specifying the elements necessary for describing depression. The features extracted from the data are then used to train the classification model, which is done using several machine-learning techniques. The decision stage uses a trained model to classify patients as happy or unhappy based on their health. Machine language and sensor data are utilised to track mental illnesses such as depression, anxiety, and bipolar disorders. 

The requirement for therapy is frequently not met in the later stages, according to the World Mental Health Survey Consortium, which finds that industrialised countries have more mental health patients than less developed ones [1]. A multi-dimensional Bayesian network classification technique, known as the MBC technique, was used to examine the contemporaneous identification of hopelessness and co-occurring mental illness [3]. In an experiment, significant sad and happy patients were utilised, along with high-risk unhappy patients, to measure excitation-based dialogue metrics such as the glottal and voiced jitter flow spectrum. Vocal jitter is a good indicator of frequency instability, and the glottal flow spectrum shows how airflow impacts the spectrum [4]. The researchers suggested an “on-body” device to monitor MDD and evaluate available treatments. They used a database containing patient phone calls captured while the patients were in the office. The study evaluated the patient’s level of depression using the Hamilton Depression Rating Scale (17 items, HAM-D) [6]. Another researcher applied the idea that free speech, as opposed to recorded speech, is a better way to describe clinical pain. Utilising the support vector machine model, they spread the cross-approval technique known as “leave-one-out cross-validation” (SVM). Using an open-source programme called “open SMILE,” a small number of low-level descriptors (LLDs) that can be viewed as edge-by-edge descriptions were selected. Since it was believed that SVM provided a better order, the general acknowledgement velocity of unfettered speech was anticipated to be faster than that of reading discourse [7]. The experts proposed a framework in which they eliminated the acoustic highlights of young adult patients and then, using two different AI techniques—the Gaussian mixture model (GMM) and the support vector machine model—divided the remaining data into two distinct classes, the discouraged class and the control class (SVM). Component extraction was applied to the speech data set provided by the Oregon Research Institute, which contains the sound diaries of 139 young people. 

To clearly show the disparities in the discourse of discouraged and controlled patients, 14 audio highlights were chosen. Numerous studies were conducted using a combination of various highlights and AI methods on male and female patients; the average characterisation accuracy for male patients was 83%, while that for female patients was 75% [5]. Another expert presented the framework to separate individuals deterred by a relative inquiry by including a choice approach and obtaining the top K highlights. They used a two-stage included determination approach by merging the insignificant repetition maximum with the order of them into channels, coverings, and implanted arrangements for their highlight selection (SFFS). The second phase entails figuring out which collection of abilities will enable one to assess the seriousness of a challenging issue and even forecast future results through follow-up testing. The third step is to choose the best communication technique because the doctors have successfully found an emotionally supportive network. The K-mean and the support vector machine (SVM) model were recently employed to carry out the order [8,9]. Component determination measures a very efficient pursuit calculation when required, which generates considerable computational expenditure, and information gathering measures their combined subjects to comprehend sections, image portrayals, and meetings. Another researcher created an approach to recognising depression using speech and facial expressions. The following provides an example of the system. Cutoff points on the BDI-II were utilised to come to a conclusion, and both video and audio features were chosen using principal component analysis (PCA) [10]. 

The researcher also discussed creating a chatbot to analyse user voices to detect whether they were depressed while identifying the causes of unhappiness by using a radial bias function network to determine the cause. Other studies involved physically collecting data or using a company (such as DVAC) to do so, preprocessing the data, selecting features (such as prosodic, glottal, spectral, TEO, and cepstral features), and then classifying the data using mathematical techniques and algorithms such as SVM, K-mean, fivefold cross-validation, and regression [19]. Reading a paragraph, looking at photos, and doing interviews were all part of the data collection process; speech and video data are gender-specific. Different strategies were discussed and implemented, and each had its result. The initial method was analysing voice sample data collected from lifeline numbers [11]. The K-mean approach is another option. Although it produced results in the right direction, it was “tough to quantify and monitor” [12]. A neural network model that could depict the degree of sadness was created by learning to recognise “red alarm signals” [13]. Despite its effectiveness, a logistic regression model was biased against men [14]. The final solution depended on a BDI questionnaire and speech recognition using a combination of K-mean and Google API. Still, it had the drawbacks of poor accuracy and dependence on the questions [15]. A downturn-related development unconnected to the other parts of the assessment and not counted in the downturn scale might be a fraction of language. Investigating whether the observed verbal movement represents the presence or absence of mourning in a person’s current emotional condition might also be noteworthy (for example, burdensome attributes). Another thing to think about is whether low language mobility indicates a problematic situation in the present or something that separates those who are prone to melancholy from others who are not (e.g., non-burdensome characteristics). Because self-announced wretchedness varies, the algorithm can calculate the BDI score based on the volume of annoying side effects and the severity of mental illness [16,17]. 

To the best of our knowledge, there has not been any research on the use of linguistic abilities to identify depression-based language. However, language work allows us to computerise the diagnosis of sadness and expand screening capacity because voice tests and questionnaires can be completed. Speech may be used to prevent and treat melancholy. In the future, we hope to create a comprehensive voice biomarker for depression that will help doctors diagnose depression in patients with a range of mental illnesses [18,20]. Thirdly, this study’s fascinating results imply that intricate cerebral availability attributes might precisely depict each individual’s thought process while determining melancholy. The early detection of demoralisation for medical therapy may profit greatly from simple measures to detect undesirable side effects in daily life. A reliable predictor of psychological health and alexithymia is the presence or absence of grief’s side effects in individuals with various mental illnesses [21,22]. It is particularly fascinating to look at people with PD, the most common mental illness in the US. This data set demonstrates how dopaminergic neurotransmitters contribute to depression in PD patients. Even though motor symptoms are a reliable indicator of the beginning of dopamine therapy, depressive symptoms are much more common in PD patients than in healthy controls, demonstrating that PD and depression play a crucial role in the early detection and treatment of depression. Everyone anticipates suffering, but we do not realise that it may coincide with a dismal time. An individual’s emotional state of sorrow can impact the acoustic qualities of speech. However, it is still unknown how important acoustic highlights are for the early recognition of melancholy and, more specifically, the discovery of sadness. Sadness can happen to anyone or any character and usually produces a milder condition than depression [23]. On one level, it is unsurprising that a high risk of extreme unhappiness is inherited and that severe manifestations are significantly correlated with this risk. It appears that these characteristics are influenced by similar hereditary factors because there is a correlation between variations in ventral hemisphere volume and the risk of experiencing sporadic severe sadness. 

This relationship helps explain how melancholy develops into psychological instability. However, even while this is not necessarily depressing, it does imply that they have some characteristics in common that are influenced by a similar hereditary component [24]. One could argue that the apparent connection between severe manifestations and a family history of excessive pessimism is not surprising. Indeed, earlier studies have indicated that individuals with depression tend toward scepticism, which may account for some of this improvement. The majority of developed frameworks employ one of two techniques, with the exception being voice-based programmed grief detection. In this work, we use a direct relapse model to predict the intensity of grieving, and we find that fundamental relapse models dramatically increase the severity of grief in practice. We also employed the STEDD-20 model, which, depending on language and emotion, is the best tool for recognising sadness in a comparable data set. This model generated a consistent BDI score.

The Hamilton Anxiety Scale indicates that it is challenging for patients with sound subjects and wretchedness to comprehend and articulate their sensations. According to the PERM scale, it would be difficult to distinguish between sentiments, think remotely, express emotions appropriately, and do things in a theatrical or jittery manner. The dramatic or jumpy PERM styles did not predict difficulties in distinguishing feelings, but the solo PERM style and the PERM-subordinate style of superior subjects did. It has also been demonstrated that individuals with ADHD frequently have hyperactivity, carelessness, diminished compassion, and a predisposition to injure themselves. Aside from other symptoms, it has been shown that those with ADD/ADHD frequently exhibit hyperactive behaviour, extreme imprudence, hyper-forcefulness, low confidence, impotent restraint, and considerable degrees of anxiety, grief, discomfort, or wretchedness.

## 3. Materials and Methods

The model was trained using the AVEC-2019 dataset by the design methodology. Audio recordings of depressed patients conversing with an AI assistant during their recorded sessions are included in this dataset. The age ranged from 16 to 64 years, with 32.5 years being the average. The recorded sample duration varied from 8 to 23 min, with an average recording time of 18 min. In total, 170 recorded samples were used. We preprocessed the collected segments to extract the audio file. We only kept the portion of the transcript file that contained the sad person’s voice and discarded the rest using a voice activation detection technique and the MATLAB toolkit. After extracting the usable portion and cleaning the dataset, we created two sets of audio features. We used an open-sourced tool called open SMILE to extract the features from the dataset. The first set contained statistical elements for descriptors of the lower level, while the second group had the cosine coefficients for discrete transformation for each descriptor in the audio segment. We reduced the complexity of the estimated features by preserving the coefficients from the second set and normalising the features from the first dataset. All 3300 characteristics were retrieved, 35 of which had to do with spectra, mass, and energy and included things such as loudness, harmonics, and skewness. 

Whenever the analysis is made to observe the depression characteristics of an individual, it is a significant task to avoid all hidden networks in the network. Therefore, if CNNs are incorporated, then all hidden characteristics of the audio features must be removed from the system, and, as a result, the unfilled state is filled using noise factors. Hence, to avoid noise characteristics in the proposed detection method, random forest is incorporated with a set of decision variables, where both the recession and classification of audio states are processed. Since the proposed audio device is based on a set of generalisation features, a good prediction technique is needed; thus, random forest is introduced, with high predicting accuracies. Furthermore, all the high-level components in random forest provided precise event handling technology by using the desired event name. Therefore, random forest can easily handle large audio dataset features by utilising the entire node set at the correct time periods. Jitter, F0 score, shimmer, including their cosine coefficients, and Mel-frequency cepstral coefficients were the ten elements, and they were all associated with acoustic and vocal qualities. We generated the dataset randomly, developed feature selection and feature ranking algorithms, and then selected and ranked many vital qualities according to their value and priority. For training, testing, and validation, we split the database into three equal groups, 80:10:10. We employed Mel-frequency cepstral coefficients to assess or classify pitch-related content for a better classification than other factors. We used a genetic algorithm to enhance the efficiency of categorisation, visualisation, and selection for the attributes gathered from the dataset. There were no spectrograms in the dataset. The argumentation excerpts were skipped by one second when the audio files were initially cut into seven-to-ten-second segments. 

We performed segmentation by calculating the average of the right and left channels. The amplitude and frequency ranges were also restricted to 15 kHz, and normalisation was performed by mapping the minimum and maximum values between −1 and 1. Using the Pysox audio manipulation toolkit, we sampled and segmented audio recordings according to their period, getting acoustic samples while disregarding background noise. After segmenting the speech samples, we produced a spectrogram for a particular voice sample and then trained and validated convolutional neural networks on it. 

### Feature Extraction from Audio Segments

We first used data preprocessing techniques on the dataset to adapt it to the requirements of our model, as depicted in Figure 1 and Figure 2. After segmenting the audio data into digestible bits, we utilised dimensionality reduction to draw deep features from the dataset. We compress the dimensionality of the input parameters into feature vectors to avoid utilising unnecessary memory. We used a victimisation regression strategy to capture the dynamic data through the feature vector while reducing their spatiality in order to generate a sadness scale. After fragmenting the audio clips and determining their period grammatical spectral estimates, we converted them into spectrograms. The Mel-frequency cepstral constant (MFCC) and combined audio characteristics were extracted from the resulting spectrogram using the deep feature extraction technique. For preprocessing in a deep characteristic style, the material facts for each pattern were split into short audio segments. The suggested segments were resized and removed. The generated components were subsequently fed into a deep network to extract the relevant properties. We ranked and normalised the features in line with the FDH set rules of patterns by converting the ways into 0s and 1s. The output was a single row of a vector. We used pre-trained convolutional neural networks that used residual learning methods in this design. 

We tweaked the boundaries of a ready-made ResNet architecture to get the classifier ready. We employed a tiering methodology in which the peripheral layer of the design is replaced with the layer of appropriate measures indicated by the dataset. In this model, the eighth layer of the fully convolutional network is changed to a new layer that contains two classes, discouraged and non-discouraged, with yields equal to the number of class forecasts and frozen layers being the pre-made ResNet designs. We employed ResNet-50 engineering to extract highlights from the sound dataset. Convolutional networks with many layers and fifty-five phases make up the ResNet-50 architecture. Each convolutional square and personality block consists of three convolutional layers. We fit the pre-prepared design to our sound dataset by employing two hyper-boundaries for learning the rate and the number of completed ages. To measure our learning rate, we kept the number of periods as a single pass over the dataset and set the defined incentive’s beginning value to 0.01 or 0.001. 

By fine-tuning the hyper-limits, the classifier can gain features at the irrefutable level by changing the model with the dataset during preparation, which is difficult while building the model regularly. We altered the dataset using a stochastic angle plunge and restarted the calculation. We recently processed the initiation reserve and improved the information argumentation to set up the convolutional neural organisation. When the value of unlucky effort is diminished, we find the incentive with the highest learning rate. We balanced and froze each convolutional layer except the final one. We trained the last layer using actuation values that had recently been established. The cycle length and information argumentation were used as one boundary as we introduced the final layer with multiple ages. The frozen convolutional layers were thawed once the last layer had been prepared, and the learning rate for the first layer was decreased by three to ten compared to the previous layer. We again determined the rate of the learning incentive, where the estimation of terrible tasks is continuously reduced. We trained the whole convolutional neural network with cycle multiple boundaries, spaced by two, until it was over-fitted, as illustrated in Figure 3.

## 4. Results

Even if social media provides a tool to track someone’s current mental state, a person’s feelings or thoughts might occasionally be influenced by one or more indirect factors, so this information cannot be used only for diagnosing depression. As a result, we used the AVEC-2019 dataset to detect depression from acoustic signals. In addition to thorough questionnaire responses, audio and video recordings were also gathered as data. The data extracted from the AVEC dataset was transcribed and annotated to note any deviations from the usual verbal and nonverbal elements. The 2019 Audio/Visual Emotional Challenge and Workshop’s AVEC-2019 dataset, which has been further processed by USC’s Institute of Creative Technologies and shared in part, includes all the audio sessions recorded, along with supplementary information and relationship metrics (AVEC 2019). 

The data were divided into 11 distinct folders for training purposes, as shown in Table 1. After each folder receives its unique model training, the overall results are averaged for testing purposes. Only 10% of the randomly selected data from each patient was used for training. The data types have also been modified from a 64-bit float to a 32-bit float. Each created folder has enough RAM for training because each model’s data frame is removed after training to make room. The data were preprocessed to remove irrelevant rows if 50% or more of the data were zero. The dataset had about 190 recorded sessions, with a total length of 8 to 35 min and an average of 17 min. As a result, an unequal dataset could produce distorted results. A reoccurring finding was that some traits that people emphasise might only apply to them because of individual variances in characteristics or personalities. It was found that participants with non-depressed class labels were more frequently seen than participants with depressed class labels. We used sampling to sample and reorganise the asymmetric dataset. A correlation matrix is developed to identify the relationships and potential interactions between the various audio components. The correlation coefficient values that were obtained vary from 0 to 0.4. 

The dataset contains 189 sessions. The recorded audio recordings from the computer-based interview session were included in the AVEC dataset. Throughout the session, we extracted the features from the audio dataset at 12 ms intervals using the COVAREP toolbox from Github. We used feature selection on the retrieved parts to determine which features would influence the dataset. The features were F0, NAQ, QOQ, H1H2, PSP, MDQ, peak slope, Rd, Rd Conf, MCEP 0-24, HMPDM 1-24, HMPDD 1-12, and Formats 1-3. The format file, total time, and speaking time for each participant were all included in the transcript file. Rows with 50% or more values set to zero have been removed from the data by preprocessing since they are meaningless. Additionally, as shown in Figure 4, a BDI-II score column is added to each file for the model’s training. Figure 4 deliberates the region of operation for the receiver, which is specified within the defined area of 0.48 m where the audio device operation is performed. The designed audio device usually operates with two different rates, which are indicated as false and true samples; thus, in accordance with the defined limit, the receiver operates without failure margins. It is also specified that the marginal rate is maintained for all the algorithmic cases and not specially provided to CNNs or random forest. However, in the proposed method, the characteristics of the receiving device are checked only with the defined characteristic curve, which varies at some points above the defined rate. The major reason for such characteristic variations is the presence of the noise factor, and it will be further reduced by providing better training of all audio samples before prediction. Additionally, in Figure 4, no poor performance is found for the designed device, and only a low false rate is maintained until all samples in the intellect are detected.

Figure 5 shows the feather values of error representations that are present in existing and proposed audio training features, which are simulated using best feature values. In the common measurement set, the feature values are changed from 10 to 100, and within the defined range, the best feature values are chosen as 20, 40, 60, 80 and 100, respectively. Since the number of audio measurements is increasing with frequency, the error rate, which is measured using the root mean square and absolute values, is maximised. Further, in the comparison state, it is observed that the error values of the proposed method are much less, thus minimising the sensitivity of the audio features in the system. This can be verified using the best feature of 60, where the state of an individual under depression is observed with an error of 11% and 9% for the existing and proposed methods, respectively.

Figure 6, Figure 7, Figure 8, Figure 9 and Figure 10 show how distinct each feature is from the others. Additionally, the impact of every characteristic on the factor used to forecast a score is looked at. In contrast to the proposed model, we predicted the BDI-II scale for the test individuals using a random forest regressor with 40 estimators. When figuring out how accurate the model is, it is also assumed that someone with a depression scale value is depressed, even if they are not depressed in other ways. A sad person is referred to as “1” in the newly added binary classification column. We evaluated the model’s performance by comparing categorisation and prediction similarities using the readily available participant labels. We simultaneously did a manual investigation and a machine investigation. We considered a response to be affirmative if the question was answered “yes” in the recorded session, and the model also offered improved precision for the same class. A negative response emerges from any dispute or debate over the categorisation. We computed the root mean square error and average mean error for calculating the model loss when projecting the BDI-II scale for a patient.

The algorithm that performed the best was found to be random forest, which had a mean average error of 8.4235 and a mean error of 8.5696. To forecast the depression scale, we incorporated the characteristics of handwriting, audio, and art samples. The effectiveness of the random forest algorithm has been carefully examined. The technique improves model precision by reducing over-fitting in decision trees. It supports the depression class classification and prediction problems and the BDI-II scale. The method in the dataset supports both continuous and categorical values. If the dataset is inconsistent or lacking, the random forest technique is used to preprocess the dataset by adding actual values. Because the algorithm uses rule-based methodology, dataset normalisation is not necessary. Specificity, sensitivity, accuracy, and precision values for the random forest algorithm’s classification and regression results on the handwriting, drawing, and speech samples were 86.13%, 86.55%, 88.97%, and 87.46%, respectively (Table 2). The accuracy was determined to be 87.56% for the anxiety or stress class for scores between 0 and 13; 88.74% for the mild depression/anxiety class for scores between 14 and 19; 87.3% for the moderate depression/anxiety class for scores between 20 and 28; and 89.45% for the severe depression/anxiety class for scores between 29 and 63.

We examined and assessed the individual research for the bulk of the methodologies and architectural performances using the AVEC-2019 dataset. The task forecasts the depression score using the BDI-II scale by examining fluctuations in the patterns visualised based on the recorded sessions in the dataset.

We divided them into three equal groups to conduct training, testing, and validation on the recorded sessions. We used supervised-based learning methodologies for training and validation and unsupervised ones for testing. Several machine-learning methods were applied to the dataset to choose the algorithm with the best accuracy. Random forest was the model that performed the best on the dataset. The random forest technique showed accuracy using the training and testing datasets, with few model losses. Table 3 and Figure 11 and Figure 12 display the model loss produced by the random forest algorithm, along with a summary of the outcomes of the random forest approach.

## 5. Conclusions

This study has developed an architecture for BDI-II scale prediction and depression classification using audio samples. Using the AVEC-2019 dataset, we used audio samples to train the model. This dataset contains audio recordings of depressed people conversing with an AI helper in recorded sessions. We took audio samples from the sessions that had been recorded. After segmenting the audio data into digestible bits, we utilised dimensionality reduction to extract deep features from the dataset. We only kept the portion of the transcript file that contained the unhappy person’s voice and discarded the rest using a voice activation detection technique and the MATLAB toolset. One of the primary developments for understanding the depression characteristics of an individual by using a set of audio features is saving the life of the individual before they enter into a perilous resolution. The projected model is designed with a larger amount of input audio data, which is processed using a five-stage process. In addition, a frequency-varying system was developed for appropriate spectrogram measurements; hence, large audio features are converted to smaller sample sets for further processing. Moreover, the proposed method is incorporated in all situations where concurrent audio features are extracted. During audio feature extraction, the device is allowed to perform under a curve region that is at 0.8 m from the body area; thus, various kinds of radiation are avoided. As the region of operation for the receiver is set at fixed values, only the best iteration values are considered, where both mean square and absolute errors are measured. In the comparative measurement process, it is observed that the proposed method, with network parameters such as sensitivity, specificity, and accuracy, proves to be much more effective as the audio samples are appropriately decoded in the output unit. The random forest method was the best-performing algorithm, with the accuracy and precision of 88.23% and 87.46%, respectively. To forecast the depression scale, we incorporated the characteristics of handwriting, audio, and art samples. Additionally, we predicted the BDI-II scale for depressed people using various machine-learning techniques and compared the results. The algorithm that performed the best was found to be random forest, which had a mean average error of 8.4235 and a mean error of 8.5696. Hence, we may conclude that by utilising audio sample features, we can effectively predict the depression scale. However, the primary limitation of the projected model is that if any algorithmic parameter other than the depression state is tested, then the output characteristics change in a complete form, and thus, complete knowledge about inducements is not captured. However, in the future, the proposed work with audio segments can be extended to provide support to all types of medical-related identification systems by using sample test systems.

## Figures and Tables

**Figure 1:** Audio segments converted into a spectrogram consisting of audio features.

**Figure 2:** Feature extractions for audio samples.

**Figure 3:** Network architecture for ResNet-50 classifier.

**Figure 4:** Receiver operating characteristic curve for depression detection using audio segments.

**Figure 5:** Comparison of RMSE and MAE with best features.

**Figure 6:** RMSE and MAE for RNN-C3D NAQ.

**Figure 7:** Comparison of RMSE and MAE for C3D QOQ.

**Figure 8:** Comparison of RMSE and MAE for RNN-C3D.

**Figure 9:** Comparison of RMSE and MAE for C3D H1H2 and PSP.

**Figure 10:** Comparison of RMSE and MAE for RNN-C3D MCEp 0-24.

**Figure 11:** Training and testing accuracy using random forest.

**Figure 12:** Model loss using random forest.

**Table 1:** Performance of the Deep Net feature on the development set and the test set in a dataset for audio segments.

Partition	Methods	Segment Type	RMSE Score	MAE Score
**Training**	**Deep Learning (Proposed)**	Waveform	9.2589	6549
		Spectrogram	10.0124	8523
**Testing**		Waveform	11.2365	3698
		Spectrogram	9.4589	1278
**Training**	**Meta-Heuristic (Existing)**	Waveform	8.5	6.43
		Spectrogram	9.1	6.21
**Testing**		Waveform	9.7	7.47
		Spectrogram	8.4	7.80

**Table 2:** Extracted features for the audio dataset from the AVEC-2019 dataset.

Methods and Metrics	RMSE (Proposed)	MAE (Proposed)	RMSE (Existing)	MAE (Existing)
C3D F0	10.68	8.46	11.21	10.4
RNN-C3D NAQ	10.94	8.40	11.86	10.9
C3D QOQ	10.86	8.76	12.42	10.3
RNN-C3D	10.67	8.69	12.51	10.12
C3D H1H2 and PSP (2 models)	10.45	8.34	12.22	10.96
RNN-C3D MCEp 0-24 (2 models)	10.91	8.23	12.14	11.24

**Table 3:** Sensitivity, specificity, precision, and accuracy values using a random forest classifier.

**Folds**	**Performance Metrics (Proposed)**			
	**Specificity**	**Sensitivity**	**Accuracy**	**Precision**
**Fold-I**	0.8954	0.8869	0.8832	0.8971
**Fold-II**	0.8756	0.8874	0.8730	0.8945
**Fold-III**	0.8631	0.8656	0.8834	0.8764
**Fold-IV**	0.8807	0.8723	0.8954	0.8821
**Overlapped**	NULL	NULL	NULL	NULL
**Depressed**	0.8754	0.8565	0.8625	0.8752
**Non-Depressed**	0.8682	0.8609	0.8771	0.8721
**Average**	0.8613	0.8655	0.8897	0.8746
**Folds**	**Performance Metrics (Existing)**			
	**Specificity**	**Sensitivity**	**Accuracy**	**Precision**
**Fold-I**	0.943	0.992	0.890	0.934
**Fold-II**	0.921	0.876	0.909	0.999
**Fold-III**	0.990	0.929	0.923	0.895
**Fold-IV**	0.901	0.911	0.946	0.916
**Overlapped**	2	4	3	4
**Depressed**	0.905	0.943	0.967	0.928
**Non-Depressed**	0.899	0.902	0.978	0.942
**Average**	0.891	0.995	0.981	0.986

## Data Availability

The data presented in this study are available upon request from the corresponding author.
